This article has been retracted.

# C-myc/TSPEAR-AS2 Axis Facilitates Breast Cancer Growth and Metastasis in a GLUT1-Dependent Glycolysis Manner

**DOI:** 10.1155/2022/4239500

**Published:** 2022-06-03

**Authors:** Jian Xu, Tao Li, Yang Zhang, Donghai Qiu, Nan Chen, Xupeng Chai, PengLi, Jia Li

**Affiliations:** ^1^SAN Biomedical Center-Zhejiang SAN Biomedical Technology Co., Ltd., China; ^2^Sino-American Cells Biotechnology Co., Ltd., China; ^3^Suzhou Institute of Biomedical Engineering and Technology, Chinese Academy of Sciences, China; ^4^Department of Cardiac Surgery, Zhongshan Hospital, Fudan University, Shanghai, China; ^5^Institute of Orthopedic Research, Zhejiang University, Hangzhou, Zhejiang 310000, China; ^6^Department of Anesthesia, The Sixth Medical Center of Chinese PLA General Hospital, Beijing 100048, China; ^7^Department of Nutrition, Jinhua People's Hospital, China

## Abstract

A large number of facts have shown that epigenetic modification and metabolic reprogramming represented by noncoding RNA play an important role in the invasion and metastasis of breast cancer, but the mechanism is not clear. The purpose of our study is to find a new biomarker of breast cancer and to provide a new perspective for regulating glucose metabolism and aerobic glycolysis of BC. In this paper, by downregulating C-myc protein, our team found that the expression of long-chain noncoding RNATSPAR-AS2 was significantly downregulated. However, the expression of long-chain noncoding RNASPAR-AS2 in BC is relatively high, and the prognosis is poor. TSPEAR-AS2 can promote the malignant phenotype of BC cells, including proliferation, apoptosis, invasion and metastasis, and glycolysis. At the same time, TSPEAR-AS2 can also upregulate the expression of GLUT1, an important regulator of glycolysis, thus promoting the metabolic reprogramming of BC. Molecular mechanism experiments show that TSPEAR-AS2 may promote the expression of GLUT1 by participating in IGF2BP2 modified by the GLUT1 gene. Our results suggest that the C-myc/TSPEAR-AS2/GLUT1 axis promotes the invasion and metastasis of BC by inducing glucose metabolism reprogramming. However, more phenotypic and molecular mechanism results need to be further verified.

## 1. Introduction

Breast carcinoma (BC) is the first diagnosed malignancy and the second female death reason globally. Sustaining proliferation has been demonstrated as the most common characteristic of BC [1]. Some scholars have developed targeting drugs for promoting BC-related molecules, but because BC has obvious heterogeneity among different individuals, the schemes for these protein molecular targets are prone to problems such as target loss and mutation drug resistance, which greatly limit the clinical application of this strategy. Thus, it can be noticed that more broad-spectrum, more conservative, and higher-dimensional interventions may achieve better results. The survival of a tumor is inseparable from energy supply, and the metabolic capacity and characteristics of a tumor directly determine the energy acquisition and biological supply of cancerous cells. Therefore, the study on neoplasm metabolites has rapidly become a new research hotspot.

lncRNA is a novel form of nonprotein coding RNA > 200 nucleotides [2]. Recently, a number of lncRNAs have been identified, which take part in the regulatory network of hematopoietic malignancies [3]. In fact, numerous lncRNAs have been identified to be cancer repressors or tumorigenesis in investigations, because they directly or indirectly regulate the expression of genes related to tumor formation, development, and chemotherapy resistance [4]. For instance, long-stranded noncoding RNAHOXB-AS3 is capable of modulating ribosomal RNA transcription in NPM1-mutated acute myelocytic leukemia [5]. Additionally, acute myelocytic leukemia can progress faster when MIAT is present through negative regulation of miR-495 [6]. Long-stranded noncoding RNAGAS5 regulates the tumorigenesis and metastasis of human B-lymphoblastic leukemia by sponge absorption of miR-222 [7]. Recently, TSPEAR-AS2 has been found to promote drug resistance and myeloma cell growth and has been found to enhance cell growth and drug resistance through p38 and JNKMAPK pathways [8]. However, the inherent importance and function effect of TSPEAR-AS2 in the development of BC is still greatly unclear.

Cancer cells absorb glucose under aerobic conditions and convert it into lactic acid, which is called the Wahlberg effect [9]. Sufficient quantities of ribotide, proteins, and lipids extracted from this glucose metabolism are necessary for the rapid growth and cancerous cellular fission [9]. Activation of the Warburg effect is a process that involves the upregulation or downregulation of many rate-limiting enzymes [10]. Targeting Warburg effects has become an important part of antitumor treatments, for instance, hypoxia-inducible factor 1 (HIF-1) is considered a novel treatment option in JAK2V617F-positive myeloproliferative malignancies [11]. However, the underlying mechanism for initiating and promoting the Warburg effect process in BC is still unknown.

Compared with normal cells, the reprogramming of tumor glucose metabolism is mainly characterized by a remarkable increase in the metabolic activity of aerobic glycolysis, resulting in the accumulation of lactic acid and other acidic substances, which promote the malignant phenotype of the tumor directly or indirectly, including proliferation, antiapoptosis, and chemotherapy resistance [12]. In addition, glucose metabolism reprogramming can increase the EMT process to promote tumor metastasis [13]. Therefore, there is a close relationship between glucose metabolism reprogramming and BC invasion and metastasis. Glucose metabolism reprogramming promotes the invasion and metastasis of BC, but the specific regulatory factors and pathways of glucose metabolism reprogramming in BC are still unclear [14].

We indicated that TSPEAR-AS2 was remarkably enhanced in BC cellular lines. The functional loss test showed that it had tumorigenic effects on the growth, invasion, and aerobic glycolysis of BC cells. Mechanistically, TSPEAR-AS2 was associated with GLUT1 mRNA and promoted its expression and stability. Further studies indicated that TSPEAR-AS2 interacts with GLUT1 mRNA in an IGF2BP2-dependent manner and positively regulates the stability of GLUT1 mRNA. TSPEAR-AS2 promotes BC through GLUT1. Our investigation not only led to the discovery of a new biomarker for TSPEAR-AS2 but also provided a new perspective for regulating BC glucose metabolism and aerobic glycolysis.

## 2. Materials and Methods

### 2.1. Cell Culture

Cultured human BC cell lines MDA-MB-231, T47D, BT-20, SK-BR-3, and MCF-7 were purchased from the Shanghai Cell Bank of Chinese Academy of Sciences. In the RPMI-1640 medium (GIBCO, Gaithersburg, MD, USA) containing 10% heat-inactivated fetal bovine serum (Sigma-Aldrich, St. Louis, Missouri, USA), the fluid was changed every other day. When 90% of the cells were fused, they were inoculated into a 6-well plate preplaced with cover slides, and the number of cells per well was about 5 × 10 ~ 5 and cultured in a humid environment of 37°C and 5% CO_2_.

### 2.2. Plasmids Construction and Transfection

TSPEAR-AS2 siRNA (si-TSPEAR-AS2) and negative control siRNA (si-NC) were purchased from GenePharma (Shanghai, China). The pcDNA3.1-GLUT1 (GLUT1) and pcDNA3.1-control (vector) were harvested from GeneCopoeia (Guangzhou, China). Lipofectamine 3000 (Life Technologies Corporation, Carlsbad, CA, USA) was used for transfection, which was done according to the manufacturer's guidelines.

### 2.3. Quantitative Real-Time PCR (qRT-PCR)

The cells were inoculated in Petri dishes, and the cell density was adjusted to 1 × 10^6^ cells per dish. After the cells were attached, different doses of curcumol were added. The cells were collected 48 hours after administration, and total RNA was extracted by adding TRIzol reagent, chloroform, isopropanol, and ethanol in turn. Total RNAs were isolated using RNAiso Plus Kit (Takara, Kusatsu, Japan). In addition, total RNAs were reversely transcribed into cDNA using the miScript II Reverse Transcription Kit (Qiagen, Valencia, CA, USA). qPCR was carried out using the SYBR Green qPCR Master Mix (Thermo Scientific, Rockford, IL, USA). GAPDH was employed as an endogenous control, and primers used in this qRT-PCR were given as follows: TSPEAR-AS2: 5′-AGCGAAGTCCCGAACGACGA 3′ (forward), 5′TGGGCATTTCCAACGGGCCAA-3′ (reverse); GAPDH: 5′ATGATGACATCAAGAAGGTGGTG3 (forward), 5′CCATGAGGTCCACCACCCTGTTG-3′ (reverse); and GLUT1: 5′CGCGCACAATCCCTACCCATCGCC-3′ (forward), 5′-CTTCCAGAGGAGAGAGTTGGTTCTG-3′ (reverse).

### 2.4. Cell Proliferation Assay

A cell counting kit-8 assay kit (CCK-8, Beyotime, Beijing, China) was adopted to examine the cell growth curves of BC cells. The cells (2000 cells per well) were transferred to 96-well plates. The plates were cultivated at the temperature of 37°C with 5% CO_2_ for 1, 2, 3, 4, and 5 days. Within the specified time, the cells were subjected to CCK-8 solution (10 ml/well) for 2 h followed by the determination of the OD value at 450 nm. The experiment was carried out three times repeatedly.

### 2.5. Apoptosis Assay

Apoptosis staining kits (BD Biosciences, NJ, USA) were used to detect death by flow cytometry. The cancerous cells and supernatant were collected, centrifuged at 1500 rpm and 5 min, and washed with PBS. Resuspended cells were combined with Annexin-V-PE and 7AAD inside the PBS solution. The cells were placed into a flow tube and cultured in the dark at room temperature for 20 minutes. The specimens were measured by flow cytometry (FC500 MPL, Beckman Coulter).

### 2.6. Western Blot Assay

The cells were lysed with RIPA buffer, and the concentration of protein was measured using the enhanced chemiluminescence kit (Thermo Scientific, USA). The cell lysates were separated by SDS-PAGE and transferred onto a PVDF membrane, which was blocked in buffer and incubated with primary antibodies. After that, the PVDF samples were incubated overnight with secondary antibodies before being detected using an Easy Blot ECL kit (Sangong, Songjiang, Shanghai, China). The antibodies of GLUT1 and *β*-actin were obtained from Abcam (Pudong, Shanghai, China).

### 2.7. Subcellular Fractionation

In accordance with the PARIS KIT methodology, BC samples were centrifuged for 5 minutes to obtain the nucleus and cytoplasm fractions (Invitrogen). GAPDH, TSPEAR-AS2, and U6 expression levels were measured using the qRT-PCR technique.

### 2.8. Glucose Consumption, Lactate Production and ATP Generation Assay

BC cells were seeded in a 96-well plate, and the supernatants of culture media and cells were harvested separately for measuring the glucose metabolism and lactate production. Glucose uptake levels were assayed using a Glucose Uptake Assay kit (BioVision, Milpitas, CA, USA). The lactate was measured by lactate assay kit II (BioVision). The ATP generation was detected by the ATP Colorimetric Assay kit (BioVision) in accordance with the protocol of the manufacturer.

### 2.9. Extracellular Acidification (ECAR) and Oxygen Consumption Rate (OCR) Assays

ECAR and OCR were measured by the Seahorse XFe 96 Extracellular Flux Analyzer (Seahorse Bioscience, North Billerica, MA, USA). ECAR and OCR were detected by the Seahorse XF Glycolysis Stress Test Kit and Seahorse XF Cell Mito Stress Test Kit, respectively. Experiments were conducted in accordance with the protocols of the manufacturer. In brief, 2 × 10^4^ cells were plated to a Seahorse XF 96 tissue cell culture plate. After baseline assessment, for ECAR, glucose, oligomycin (oxidative phosphorylation inhibitor), and 2-DG (glycolytic inhibitor) were sequentially injected at indicated time points; and OCR was injected with oligomycin, oxidative phosphorylation reversibility inhibitor FCCP, and mitochondrial complex inhibitor rotenone + mitochondrial complex III inhibitor antimycin A (Rote/AA) at specified time points. BC data was assayed by the Seahorse XF-96 Wave software. OCR was shown in pmol/minute and ECAR in mpH/minute.

### 2.10. RNA Immunoprecipitation (RIP) and Methylated RNA Immunoprecipitation (MeRIP) Assays

RIP and MeRIP were detected by the Magna RNA-binding protein immunoprecipitation kit (Millipore) and Magna methylated RNA immunoprecipitation (MeRIP) M6A kit (Merck, Milibo), respectively, depending on their instructions.

### 2.11. Luciferase Reporter Assay

The promoter region of GLUT1 was cloned into the pGL3 plasmid. PGL3 or pGL3-glut1 and pRL-TK were transfected into BC cells, and the tspeara-as2 gene was downregulated. After 48 hours, luciferase activities were investigated by the Double Luciferase® Reporter Gene Detection System.

### 2.12. Statistical Analysis

BC statistical analyses were carried out using GraphPad 9.0 (GraphPad, Inc., USA) and presented as mean ± SD. Remarkable differences were determined by Student's *t* test or one-way analysis of variance (ANOVA). *P* < 0.05 was.

viewed as a statistical difference.

## 3. Results

### 3.1. TSPEAR-AS2 Is Upregulated in BC and Predicts Poor Prognosis

To determine the differentially expressed genes (DEGs) that occurred during the C-myc regulation, we performed a microarray to analyze the DEGs. By setting the threshold (*P* < 0.05, |fold change| > 2), the results demonstrated that TSPEAR-AS2 was significantly upregulated in BC cells (Figure 1(a)). To express the potential function of TSPEAR-AS2 in BC, via RT-QPCR analysis, we firstly detected TSPEAR-AS2 expression levels in heath breast cell line MCF-10A and five BC cell lines (BV-20, T47D, MDA-MB-468, MDA-MB-231, and MCF-7). The results revealed that TSPEAR-AS2 was highly elevated in five BC cell lines in contrast to normal cell line hFOB1.19 (Figure 1(b)). The results of immunohistochemistry indicated the expression of TSPEAR-AS2 was higher in BC compared to paracancerous tissues (Figure 1(c)). To further corroborate the clinical significance of TSPEAR-AS2 in BC patients. The Kaplan-Meier method, as well as the log-rank test, was conducted to measure the expression of TSPEAR-AS2 in the BC TCGA database, and the results indicated that BC patients with high expression of TSPEAR-AS2 were negatively associated with overall survival (OS) (Figure 1(d)). Collectively, TSPEAR-AS2 is upregulated in BC and predicts poor patient prognosis.

### 3.2. TSPEAR-AS2 Promotes the Proliferation of BC Cells and Inhibits the Apoptosis

Then we used functional experiments to verify the effect of TSPEAR-AS2 on the proliferation and apoptosis of BC cell lines. The results displayed that knocking down the TSPEAR-AS2 gene could significantly reduce the proliferation ability of BC cells (Figure 2(a)). Meanwhile, the data of apoptosis identified as well that knockout of the expression of TSPEAR-AS2 could increase the apoptosis of BC cells (Figure 2(b)). According to our findings, TSPEAR-AS2 was able to enhance BC cellular proliferation while inhibiting apoptosis.

### 3.3. TSPEAR-AS2 Associates with GLUT1 mRNA and Promotes Its Stability

Because lncRNA is involved in many biological processes, we studied the effect of TSPEAR-AS2 on BC in vitro. Furthermore, we used the Transwell assay to detect the effect of TSPEAR-AS2 on cell metastasis. The findings revealed MCF-7 and MDA/231 cells had a decreased ability to migrate after inhibition of TSPEAR-AS2 expression (Figures 3(a) and 3(b)). The above results confirmed that MAFA-AS1 was capable of improving the development of OS cells.

### 3.4. TSPEAR-AS2 Promotes the Glycolysis of BC Cells

Considering the relationship between aerobic glycolysis and tumor progression, we investigated whether TSPEAR-AS2 regulated aerobic glycolysis in BC cells. Initially, TSPEAR-AS2 knockdown of BC cells markedly reduced glucose absorption (Figure 4(a)), lactate production (Figure 4(b)), and ATP generation (Figure 4(c)). In addition, TSPEAR-AS2 knockdown in BC cells resulted in a lower extracellular acidification rate (ECAR), which is a measure of the total flux of glycolysis in cells (Figures 4(d) and 4(e)). Moreover, oxygen consumption rate (OCR), a measure of mitochondrial function, was significantly increased in TSPEAR-AS2 knockdown BC cells (Figures 4(f) and 4(g)). In general, these data strongly demonstrated that TSPEAR-AS2 was taken participated in the regulation of aerobic glycolysis in BC cells.

### 3.5. TSPEAR-AS2 Regulates GLUT1 via the IGF2BP2 Pathway

Then we analyzed the cellular location of TSPEAR-AS2 and observed that TSPEAR-AS2 was mainly distributed in the cytoplasm of BC cells, suggesting that TSPEAR-AS2 may modify downstream target genes through the posttranscriptional pathway (Figure 5(a)). Subsequently, PCR and WB experiments confirmed that TSPEAR-AS2 could reduce the mRNA and protein expression of GLUT1 (Figures 5(b) and 5(c)), while TSPEAR-AS2 could promote the stability of GLUT1 mRNA, which further indicated that TSPEAR-AS2 mediated the modification of GLUT1 through the posttranscriptional pathway (Figure 5(d)). Subsequently, RIP experiments also confirmed that there was an interaction between GLUT1 and IGF2BP2, and TSPEAR-AS2 can maintain the stability of the interaction (Figure 5(e)). Finally, through the JASPAR data, it was found that there was a C-myc binding site in the TSPEAR-AS2 promoter region, suggesting that C-myc may promote the transcription of TSPEAR-AS2 (Figure 5(f)).

## 4. Discussion

In recent years, with the comprehensive development of surgery, radiotherapy, and chemotherapy, targeting, and endocrine therapy, the therapeutic effect and prognosis of BC have made great progress [15, 16]. However, the advanced BC, especially triple-negative BC, is not sensitive to chemotherapy and targeted treatment. Furthermore, BC is prone to early metastasis, which has always been the difficulty and bottleneck of clinical BC treatment. Understanding the molecular mechanism of BC metastasis regulation is an important need to solve the bottleneck of BC treatment.

More evidence has shown that lncRNA represents an essential function in a variety of biological events such as carcinoma proliferation, migration, metastasis, and chemotherapy resistance. lncRNA ANCR induces tumorigenesis and resistance to chemotherapy in nasopharyngeal cancer via decreasing the PTEN expression [17]. In cervical cancer, upregulation of HOTAIR results in chemoresistance via promoting the HIF-1*α* expression [18]. Recently, a novel conserved lncRNA “prostate cancer-associated transcript 1” (TSPEAR Antisense RNA 2) has been characterized. Some researches have revealed that TSPEAR-AS2 was upregulated in gastric cancer, colorectal cancer, and hepatocellular carcinoma and played pivotal roles in cancer regulation [19, 20]. Recently, TSPEAR-AS2 is detected to promote myeloma cell proliferation as well as chemotherapy resistance. However, the functions and molecular pathways of TSPEAR-AS2 in BC remain uncertain. In the current research, we suggested that the TSPEAR-AS2 expression was increased in BC cells. Functionally, TSPEAR-AS2 knockdown inhibited cell proliferation and invasion. Furthermore, we demonstrated that TSPEAR-AS2 promoted BC growth and glycolysis in a GLUT1-dependent manner. Thus, our study for the first time showed that TSPEAR-AS2 promotes BC progression and glycolysis.

It has been reported that lncRNA can combine with RBPs to improve the stability of target mRNA [21]. For example, in colorectal cancer, CASC9 induces tumor growth and metastasis by interacting with CPSF3 to enhance the stability of TGF-*β* mRNAs [22]. LINC01093 links IGF2BP1 straight and inhibits the connection between GLI1 mRNA and oncogene GLI1 mRNA, causing GLI1 mRNA to degrade and inhibit HCC cell growth and spread [23]. lncRNA-assisted stabilization of transcripts (LAST) is considered to enhance the stability of CCND1 mRNA by cooperation with CNBP to combine 50 UTR of CCND1 mRNA [24]. In the present study, TSPEAR-AS2 was first validated to enhance GLUT1 expression and mRNA stability. These findings provided sufficient proof that TSPEAR-AS2 promoted BC chemoresistance by directly stabilizing GLUT1 mRNA.

Cancer cells have an abnormal metabolism characterized by strong aerobic glycolysis (known as the Warburg effect), an elevated glucose consumption rate, and high lactic acid generation [10, 25]. Emerging evidence demonstrated that the elevated aerobic glycolysis in malignancies strongly correlated with chemoresistance owing to upregulating the endogenous antioxidant capacity through the accumulation of lactate and pyruvate. Aerobic glycolysis is a promising strategy for tumor therapy [9, 26, 27]. However, whether lncRNAs are contributed to the aerobic glycolysis and resistance to drugs in BC remains unclear. Previously, 3-phosphoinositide-dependent protein kinase 1 (GLUT1) is upregulated in several human malignancies and linked to a worse prognosis [28]. Targeted GLUT1 with DAP decreased AML cell proliferation across various signaling pathways, according to a new study, suggesting that targeting GLUT1 could be a feasible therapeutic method for AML [29]. Nevertheless, the upstream regulation mechanism of GLUT1 and its function in drug resistance in BC is unclear. In the present research, knocked down TSPEAR-AS2 repressed GLUT1 and aerobic glycolysis, resulting in lower glucose utilization, ECAR, and the production of lactate and ATP, demonstrating the important part in GLUT1 in aerobic glycolysis and multidrug resistance in BC. Importantly, meRIP assays and rescue experiments confirmed that TSPEAR-AS2 mediated aerobic glycolysis by regulating the IGF2BP2/GLUT1 axis. This first finding of the TSPEAR-AS2/IGF2BP2/GLUT1 axis provides a viable strategy for future therapeutic agents targeting the aerobic glycolysis in BC.

In recent years, RNA epigenetics has now become a fascinating area of cancer research. In human malignant illnesses, M6A alteration is one of the most prevalent and essential mRNA changes [14, 30]. Some evidence indicated that the “writer,” “eraser,” and “reader” of M6A play an important part in the tumorigenesis and malignant processes. As the first eraser of M6A, IGF2BP2 is associated not only with weight gain and obesity but also with the progression of various cancers [31]. The study of IGF2BP2 and malignancy formerly concentrated on the association of IGF2BP2 single-nucleotide polymorphisms or overweight and the beginning danger of malignant tumors [32]. However, the carcinogenic effect of IGF2BP2 through mRNA demethylation has only recently been discovered [30]. New data have found that the level of IGF2BP2 is increased in AML, while in these leukemia cell lines, the downregulation of IGF2BP2 leads to an antitumor phenotype. By mRNA epigenetic modification, IGF2BP2 modulates the stability of ASB2 and RARA expressions (33). This study reveals the carcinogenic effect of IGF2BP2 via demethylated mRNA, suggesting that the block of IGF2BP2 is probably a promising cancer therapeutic protocol (33). In our study, we found that TSPEAR-AS2 promotes the stability of GLUT1mRNA in an IGF2BP2-dependent way in BC. Our results confirmed the carcinogenic role of IGF2BP2 in BC and the relationship between mRNA regulated by IGF2BP2 and BC invasion.

In summary, we demonstrated that the C-myc/TSPEAR-AS2/IGF2BP2/GLUT1 axis could regulate the aerobic glycolysis of BC cells, which modulates the sensitivity of BC metastasis. Our results provide valuable information for understanding BC metastasis and increase the possibility that targeting the C-myc/TSPEAR-AS2/GLUT1 axis may be a promising strategy to improve the efficacy of BC therapy.

## Figures and Tables

**Figure 1:** TSPEAR-AS2 is upregulated in BC and predicts a poor prognosis. (a) The results of RNA sequencing showed that the downstream target gene of C-myc. (b) The relative expression of TSPEAR-AS2 in BC cells. (c) The results of immunohistochemistry showed the expression of TSPEAR-AS2 in BC and paracancerous tissues. (d) The Kaplan-Meier plot showed the relationship between the expression of TSPEAR-AS2 and the prognosis of patients.

**Figure 2:** TSPEAR-AS2 promotes the proliferation of BC cells and inhibits apoptosis. (a) The cell proliferation of control and TSPEAR-AS2-depleted BC cells was detected by the CCK-8 assay. (b) The cell apoptosis rate of control and TSPEAR-AS2-depleted BC cells was detected by Annexin-V FITC methods.

**Figure 3:** TSPEAR-AS2 promotes the migration and invasion of BC cells. (a) The effect of TSPEAR-AS2 on the migration and invasion of BC cells was verified by the Transwell experiment. (b) The effect of TSPEAR-AS2 on the migration of BC cells was verified by the scratch test experiment.

**Figure 4:** TSPEAR-AS2 promotes the glycolysis of BC cells. (a) To determine the effect of interfering TSPEAR-AS2 on glucose uptake of BC cell line. (b) To determine the effect of interfering TSPEAR-AS2 on lactate production of BC cell line. (c) To determine the effect of interfering TSPEAR-AS2 on ATP production of BC cell line. (d) To determine the effect of interfering TSPEAR-AS2 on ECAR of BC cell line. (e) To determine the effect of interfering TSPEAR-AS2 on glycolysis and the capacity of the BC cell line. (f) To determine the effect of interfering TSPEAR-AS2 on OCR of BC cell line. (g) To determine the effect of interfering TSPEAR-AS2 on respiration of BC cell line. ^∗^*P* < 0.05 compared with the negative control.

**Figure 5:** TSPEAR-AS2 regulates GLUT1 via the IGF2BP2 pathway. (a) The subcellular localization experiment showed the localization of TSPEAR-AS2 in BC cells. (b) Observation of the effect on the mRNA expression of GLUT1 after knockdown TSPEAR-AS2. (c) Observation of the effect on the mRNA expression of GLUT1 after knockdown TSPEAR-AS2. (d) mRNA stability experiment verifies the effect of TSPEAR-AS2 on the stability of GLUT1 mRNA. (e) RIP experiment verifies the interaction between TSPEAR-AS2 and GLUT1. (f) The JASPAR database shows the promoter binding site of C-myc. ^∗^*P* < 0.05 compared with the negative control. ^#^*P* < 0.05 compared with the si-TSPEAR-AS2 group.

## Data Availability

No data were used to support this study.
